The article "Subcutaneous Fat Thickness Remarkably Influences Contact Pressure and Load Distribution of Buttock in Seated Posture" was published in 2021. Journal: J Healthc Eng.

# Subcutaneous Fat Thickness Remarkably Influences Contact Pressure and Load Distribution of Buttock in Seated Posture

**DOI:** 10.1155/2021/4496416

**Published:** 2021-11-30

**Authors:** Kuan Wang, Yufang Chen, Shangjun Huang, Lejun Wang, Wenxin Niu

**Affiliations:** ^1^Shanghai YangZhi Rehabilitation Hospital (Shanghai Sunshine Rehabilitation Center), School of Medicine, Tongji University, Shanghai 200092, China; ^2^Laboratory of Biomechanics and Rehabilitation Engineering, School of Medicine, Tongji University, Shanghai 200092, China; ^3^Sport and Health Research Center, Physical Education Department, Tongji University, Shanghai 200092, China

## Abstract

Spinal cord injury patients are prone to develop deep tissue injury (DTI) as they may spend half their time per day in sitting postures, which produce excessive load in their buttocks. However, the impact of fat thickness on the biomechanical response of buttock in sitting posture remained unclear. This study aimed to investigate the influence of subcutaneous fat thickness on the interface pressure and load distribution of buttock of seated humans. To achieve this goal, a 3-dimensional finite element model of male buttock was constructed and the contact pressure on a rigid cushion was evaluated against experimental results. The modified models, which had various fat thicknesses under ischial tuberosity, were built and used to simulate the sitting conditions with different cushion stiffnesses. In the models simulating sitting on the rigid cushion, the peak contact pressure ranges from 0.052 MPa to 0.149 MPa. In the simulation of sitting on the soft cushion, the peak stress of muscle underneath ischial tuberosity in the model with the thickest fat tissue was slightly higher than that of the other models. The results demonstrate that the fat tissue in the buttock could reduce the contact pressure when sitting on the rigid seat. However, contact pressure solely could not be used to estimate the internal tissue stress of seated buttock, especially in subjects with thicker fat tissue.

## 1. Introduction

For spinal cord injury (SCI) patients, wheelchairs are their primary mobility device. This means that they may spend half their time in sitting postures per day [1, 2]. In such conditions, buttocks are under excessive and sustained loads, which can lead to tissue deformation and make SCI patients prone to develop pressure ulcers [3, 4]. Pressure ulcers could cause pain and influence quality of life [5]. In severe cases, it could result in infection and sepsis, which are life-threatening [6]. Therefore, the prevention of sitting-acquired pressure ulcers is very important to SCI patients.

In standard seated posture, the upper body weight is transferred from lumbar spine to sacrum of pelvis, ischial tuberosity, buttock soft tissues, and finally seat surface. Thus, the tissue composition underneath the ischial tuberosity plays a crucial role in the load distribution of buttock. Gluteus muscles, subcutaneous fat tissue, and skin are major tissues around ischial tuberosity. Under loading, these tissues deformed and lead to a number of pathophysiological responses [7], which could cause superficial pressure ulcers and deep tissue injury. Unlike superficial pressure ulcers, deep tissue injury (DTI) is a severe type of pressure ulcers originating from the muscle tissue overlying bony prominences [8]. Since DTI occurs under the skin, it is hard to diagnose in an early stage. To help assess the risk of developing DTI in SCI patients, there is a need to understand the load distribution of buttock in sitting posture.

The pressure sensor is a useful tool to evaluate the interface pressure between buttock skin and seat surface. It is easily operated and could provide information about pressure distribution on the seat; thus, it is sometimes used to evaluate the risk of developing pressure ulcers and test the pressure-relieving effect of seat cushion [9]. However, the pressure sensor cannot offer the loading condition of internal buttock tissues, which prevents its further usage in clinics. By combining an animal model of DTI with computational modeling, it has been shown that direct deformation damage occurred when a strain threshold has been exceeded [10]. Therefore, the local mechanical environment within soft tissues may be a better tool to assess soft tissue injury risk.

To study the loading condition in the deeper tissue of buttock, several studies used weight-bearing magnetic resonance imaging (MRI) and compared the deformation of the buttock in unloaded and loaded sitting conditions. Sonenblum et al. [11] investigated the 3D anatomy and deformation of the buttocks during sitting in seven healthy and SCI patients, and clearly illustrated the tissue deformations through MRI images. They also studied the effect of cushion designs on the buttock deformation during sitting [12] and showed that the relationship between contact pressure and deformation varied by individuals and was highly nonlinear. Similar results were also found by Brienza et al. [13], in which they found that reductions in muscle and fat volumes in the sitting conditions varied depending on both cushion type and individual anatomy. The limitation of MRI is its time-consuming scanning process. Therefore, this method is impractical to test multiple loading conditions, e.g., sitting on seats with different cushion types, for each SCI patient.

On the other hand, finite element (FE) analysis is a powerful tool to analyze structural behavior and was commonly used to understand the response of deeper tissue of buttock. The first study quantifying the *in vivo* strain and stress distributions of subdermal tissues in sitting humans was carried out by Linder-Ganz et al. [14]. They built 2D finite element (FE) buttock models based on MRI data and found various loading conditions of the inner tissues of buttock. Makhsous et al. [15] constructed a detailed 3D FE buttock model and demonstrated that the deformation induced by sitting pressure was substantially different among muscle, fat, and skin. A sensitivity study on the materials of buttock models performed by Luboz et al. [16] showed that the stiffness of fat and muscle has an important influence on the strain variations. While these results showed that the tissue variation has a great impact on the load distribution of buttock in the sitting posture, few studies investigated the role of subcutaneous fat tissue on the biomechanics of buttock in 3D space. Although recent studies have reported the variation in the thickness of subcutaneous fat tissue of buttock [11, 13], the impact of fat thickness on interface pressure and internal stress of buttock tissues in sitting posture remained unclear.

Therefore, this study aimed to investigate the influence of subcutaneous fat thickness on the interface pressure and load distribution of buttock of seated humans. To achieve this goal, we built four 3D FE models of male buttocks with various fat thicknesses and simulated the sitting conditions with different cushion stiffnesses. This study provides insight into the prevention of DTI in SCI patients and can aid the design of better wheelchair seat cushion.

## 2. Material and Methods

### 2.1. Model Construction

We used the following steps to build the buttock FE model, which could represent a wide variety of populations. Firstly, the computed tomography images from the Visible Human Project [17] of a man were segmented using Mimics 18.0 (Materialise Inc., Leuven, Belgium), and this model was used as a template. Bone, muscle, and fat tissue in the buttock and thigh region were segmented separately. The segmentation files were imported into Geomagic Studio 11 (Geomagic Inc., Research Triangle Park, NC, USA) for further smoothing and creation of surface models. Then, these files were imported into HyperMesh 11.0 (Altair Engineering Inc., Executive Park, CA, USA) for meshing. Finally, the meshes were linearly scaled in 3D space to represent the buttock and thigh part of a man with 175 cm height, which approximated the size of the 50th percentile male [18]. The skin was offset outward from the surface of fat tissue with a unique thickness of 1.8 mm [19].

Since the buttock model was in the upright posture, it was needed to be positioned into a sitting posture. To achieve this goal, the model was assigned with material properties listed in Table 1. Poisson's ratio of the muscle and fat tissue was assumed as 0.495. Since the bone was not the major factor we want to investigate, it was treated as rigid body. Three rotational degrees of freedom were set to both the hip joints. Then, the upper surface of the pelvis was fixed, while a rotational displacement to flex the hip joint was implemented. The deformed FE model was in the sitting position (Figure 1) and served as a baseline buttock model (Model C). The model contained 474,476 elements, and the convergence study showed that this model could get the balance between simulation speed and accuracy in the calculation of stress and strain (the differences in maximum stress and strain between the current mesh and a finer mesh were less than 5%).

### 2.2. Model Evaluation

The baseline buttock model was evaluated against the results reported by Ref. [23]. Firstly, a rigid cushion model with Young's modulus of 2 GPa was built to simulate the experimental condition. The cushion model was meshed with 16 *∗* 16 *∗* 3 hex elements and has a dimension of 430 *∗* 430 mm in width and length, which was the same as the size reported in Ref. [23]. Then, the buttock model was set with a gravity acceleration of 9.8 m/s^2^. A vertically downward load of 300 N was applied to the sacrum to make sure that the total upper body weight approximated that of a 50th percentile male [24]. This load was implemented on a reference point located on the upper surface of the sacrum. The lower leg was assumed to be supported by ground or footrest of wheelchair. Thus, their weight was not considered in the model. The surface-to-surface contact was set between the skin of the buttock model and the cushion model. The friction factor was set to be 0.5 [26]. The muscle and fat were assumed to have no slipping at the interface between the two tissues. The lower surface of the cushion was fixed during all simulations. The evaluation process and the following simulation process were solved in Abaqus/Standard v6.14 (Simulia Inc., Providence, RI, USA) using static analysis.

### 2.3. Model Variation and Simulation

In the study of Sonenblum et al. [11], they reported three SCI patients with the fat thickness of 6, 15, and 30 mm under the ischial tuberosity. In this study, the subcutaneous fat thickness under the ischial tuberosity after the scaling process and flexion of the hip was about 22 cm (Model C). To cover the range of fat thickness reported by Sonenblum et al. [11], three additional buttock FE models were constructed with the fat thickness of 6, 14, and 30 mm (models A, B, and D). These models were created in the HyperMesh by morphing the surface of the baseline model while keeping the smoothness of the skin surface. The coronal views of the four buttock models are illustrated in Figure 1.

In the simulation step, the cushion model was meshed with a smaller element size (32 *∗* 32 *∗* 3 elements in total). The loading condition was the same as that in the evaluation process, except that the material of cushion was replaced by a soft one. The common stiffness of the foam in the wheelchair was reported to be 15.3 kPa [25], and this value was chosen as the material property of the soft cushion. To further test the sensitivity of cushion material property on the contact pressure and load distribution of the buttock, three other stiffnesses of the cushion (25 kPa, 50 kPa, and 100 kPa) and the rigid one (2 GPa) were also tested in the simulation (Table 1).

Therefore, four buttock models with five cushion material properties were built, and a total of 20 loading conditions were simulated in this study. For comparison of the internal load of muscle tissue, the same elements of muscle tissue within 60 *∗* 60 *∗* 60 mm cubic region underneath two ischial tuberosities were labeled in each model. The peak stress and strain of these elements were extracted and compared among 20 loading conditions. To avoid extreme outliers that may be sensitive to boundary conditions, the peak stress and strain in this study refer to the 95th percentile von Mises stress and maximum principal strain of the extracted data [27].

## 3. Results

Figure 2 shows the experimental results read off from the literature [23] and the mapping of contact pressure in our simulation of sitting on the rigid cushion in the baseline model (Model C). The contact area predicted by our model was 0.094 m^2^.

The four buttock models with different subcutaneous fat thicknesses were then loaded on the simulation condition.  Figure 3 shows the mapping of the contact pressure in the four models simulating sitting on a rigid cushion (2 GPa). The peak contact pressure ranged from 0.052 MPa (Model D) to 0.149 MPa (Model A), and the contact area ranged from 0.062 mm^2^ (Model A) to 0.100 mm^2^ (Model D). The von Mises stress and maximum principal strain of the tissue in the coronal view of the buttock are shown in Figure 4, with stress and strain concentrated on the tissue beneath the ischial tuberosity region.

When simulating the condition of sitting on a soft cushion (15.3 kPa), the peak contact pressure ranged from 0.015 MPa (Model D) to 0.020 MPa (Model A), and the contact area ranged from 0.117 mm^2^ (Model A) to 0.143 mm^2^ (Model D) (Figure 5). The stress concentration was more obvious in Model D, while the distribution of strain showed little difference among the four models (Figure 6).

In the simulation of sitting on the cushions with various stiffnesses, a minor decrease in the peak strain in the muscle underneath the ischial tuberosity could be found from the rigid cushion to the soft cushion in the four models (Figure 7). The peak strain in models A, B, C, and D was 66.73%, 64.58%, 62.39%, and 63.56% with rigid cushion (2 GPa), respectively. In the condition of soft cushion (15.3 kPa), the peak strain was 59.13%, 58.72%, 59.58%, and 60.79% in models A, B, C, and D, respectively. The peak stress also showed a decrease from the rigid cushion to the soft cushion in the four models (Figure 7). The peak stress in models A, B, C, and D was 0.0287, 0.0244, 0.0217, and 0.0224 MPa with the rigid cushion (2 GPa), respectively. In the condition of soft cushion (15.3 kPa), the peak stress of Model D (0.0158 MPa) was slightly higher than that of models A, B, and C (0.0149, 0.0145, and 0.0149 MPa).

## 4. Discussion

In this study, we analyzed the effect of subcutaneous fat thickness on the contact pressure and load distribution of buttock in the sitting posture through the FE method. Four buttock FE models with different fat thicknesses under the ischial tuberosity were built for the analysis. The results of this study highlight the crucial role of subcutaneous fat thickness in the weight-bearing of seated buttock.

The baseline FE model was evaluated in the condition simulating a sitting posture on the rigid cushion (Figure 2). The size of the model, loading condition, and material property of the cushion were set approximating that in the literature [23]. In this study, the result showed high contact pressure under the ischial tuberosity region, which is in good agreement with the mapping of the contact pressure in the literature. In other regions of the cushion, our model predicted low contact pressure, and the pattern of pressure distribution was similar to that reported by Verver et al. [23]. Therefore, the model was evaluated and could be used for further analysis.

In this study, the FE models were all created from one baseline model and all tissues except subcutaneous fat tissue were identical in the four models. This allowed us to compare the effect of fat thickness directly among the four models. In the sitting posture, we found concentrated contact pressure under the ischial tuberosity in all of the four models, whether the cushion was rigid or soft (Figures 3 and 5). Also, the von Mises stress was higher in the region under the ischial tuberosity in the coronal view of the model, which is similar to the results predicted by 2D FE models in the literature [28, 29]. In accordance with the literature, our results showed concentrated stress on the muscle directly beneath the ischial tuberosity and the fat tissue close to that region. These results indicate that the load transfer path from the upper body to the cushion would generally not be changed by the buttock fat tissue with various thicknesses.

When the subcutaneous fat was thicker, our results showed that the upper body weight distributed more evenly on the rigid cushion (Figure 3). This could be explained by two reasons: first, the model with thicker fat tissue had a larger skin surface, which increased its contact area, and second, the modulus of fat tissue is low, which means the fat tissue is more deformable than the other tissues in our model. Therefore, the thicker the subcutaneous fat tissue, the more load could be dispersed. The results of von Mises stress showed a similar trend that the models with thicker fat tissue (models C and D) had lower stress concentration on the muscle. However, Model D had slightly higher peak stress than Model C had in the muscle tissue under the ischial tuberosity (Figure 7). This result suggests that subject with thin subcutaneous fat tissue could lead to high stress in the internal muscle under ischial tuberosity when sitting on a rigid seat, but the reverse is not true. Our study confirms the results produced by Sopher et al. [29], which showed that the subjects with too low or too high body mass index could all lead to high load in the internal tissue of seated buttocks. More than that, our results suggest that an increase or decrease in the contact pressure may be not in accordance with the stress suffered by the internal muscle of buttock.

When sitting on a soft cushion, our results revealed that the contact pressure and von Mises stress were remarkably reduced compared with that sitting on a rigid cushion. The mapping of the contact pressure on the soft cushion showed that the model with thinner fat tissue caused higher contact pressure. However, the von Mises stress showed no obvious difference among the first three models (models A, B, and C), and Model D exhibited more stress concentration in the muscle and fat tissue under the ischial tuberosity region. The qualitative results of peak stress (Figure 7) demonstrated that the model with the thickest fat tissue (Model D) had the highest stress. This result indicates that the unloading effect of cushion would vary among subjects with different fat thicknesses. In this study, the soft cushion is more effective to model A in reducing stress concentration than to the other three models. Therefore, our results suggest that a soft cushion is more needed for the subjects with less fat tissue under ischial tuberosity.

The biomechanical response of buttock FE models to various cushion stiffnesses was investigated in this study. The results demonstrated that the peak internal muscle stress in the model with thinner fat tissue was more sensitive to the change in cushion stiffness. The sensitivity study also showed that the peak internal muscle stress would be reduced to a similar level when the cushion was soft enough. This result is reasonable because the thicker the fat tissue, the more capable it is to distribute loads. Thereby, the fat and cushion have a similar role in relieving internal stress. In the study of Sonenblum et al. [12] and Brienza et al. [13], the same cushion type could produce various unloading effects in different subjects. Our results reproduced the phenomena from the perspective of variation of subcutaneous fat thickness. Additionally, the results of this study suggest that the subjects with thinner fat tissue under ischial tuberosity could reduce their internal muscle stress more easily using a soft cushion.

Our findings may have several implications for the prevention of DTI. First, the results of the study indicate that contact pressure solely could not be used to estimate the internal tissue stress, especially in subjects with thick fat tissue. Second, our results suggest the important role of cushion in reducing muscle stress in the subjects with thinner fat tissue. Due to the high variability in the composition of buttock tissue among various SCI patients [11–13], using a combination of medical imaging techniques with subject-specific finite element modeling may provide insight into the optimization of an appropriate cushion for DTI prevention.

The buttock FE model we built in this study was based only on computed tomography images from a male subject. This is one limitation of this study. There are several differences in geometry and tissue composition between males and females [30]. These differences may influence the loading effect in the buttock in sitting posture. In this study, we adjusted the fat thickness in the FE model to mitigate this problem and generalize the results of this study. To fully address this problem, FE modeling based on a dataset of medical images of buttock covering both male and female subjects is needed. In this study, we used a baseline 3D FE model to create three other buttock FE models with various fat thicknesses. While this method allowed us to easily investigate the effect of fat tissue, it surely has some limitations. First, the geometry of muscle and bone structure was not changed in the four models. Therefore, the results of this study were produced by the ideal model with variation only in the fat thickness and could not represent all loading conditions in the real world. To overcome this issue, statistical models with different geometries of pelvis and soft tissues created from a dataset of buttocks should be used in the future study [29]. Second, sitting posture has a huge impact on the load distribution of buttock. Based on this model, our future research would consider the interaction between posture and geometry of seated model [31]. Third, the muscle tissue was segmented as one part in this study. In the future, more detailed segmentation of muscle tissue should be performed to produce more realistic results. Also, it is a challenge to identify the neutral state of the soft tissue in the buttock. In this study, the state of soft tissue in the seated model after changing from the upright posture was assumed to be the neutral state with no strain. Future studies could perform *in vitro* experiment to identify the neutral state of the soft tissue to further improve the accuracy of the buttock model. In addition, muscle is sensitive to pressure load [32]; thus, cell-level finite element modeling of buttock can also be the objective of future studies.

## 5. Conclusions

The fat tissue in the buttock could reduce the contact pressure when sitting on the rigid seat. Contact pressure solely could not be used to estimate the internal tissue stress of seated buttock, especially in subjects with thick fat tissue.

## Figures and Tables

**Figure 1:** Finite element models of buttock with four subcutaneous fat thicknesses and the loading condition in this study.

**Figure 2:** Contact pressure distribution in the literature [23] ((a), recorded by the pressure sensors) and our study ((b), computed by the finite element method and automatically interpolated by software).

**Figure 3:** Contact pressure in the simulation of sitting on a rigid cushion.

**Figure 4:** von Mises stress and maximum principal strain of buttock tissues in the coronal view in the simulation of sitting on a rigid cushion.

**Figure 5:** Contact pressure in the simulation of sitting on a soft cushion.

**Figure 6:** von Mises stress and maximum principal strain of buttock tissues in the coronal view in the simulation of sitting on a soft cushion.

**Figure 7:** Peak strain and stress in the muscle underneath the ischial tuberosity (the image in the bottom right corner shows the region of interest in the coronal view (black box) where we extracted the peak strain and stress from).

**Table 1:** Material properties of the buttock model.

Component	Formulation	Material	Density	References
Bone	Rigid	—	1000 kg/m^3^	[20]
Muscle	Ogden hyperelastic	*μ*1 = 1907.4 Pa, *α*1 = 4.6	1100 kg/m^3^	[20]
Fat	Ogden hyperelastic	*μ*1 = 1166.7 Pa, *α*1 = 16.2	920 kg/m^3^	[20]
Skin	Elastic	*E* = 0.15 MPa, *v* = 0.46	1100 kg/m^3^	[21]
Pelvic cavity	Elastic	*E* = 0.01 MPa, *v* = 0.49	1060 kg/m^3^	[22]
Cushion	Elastic	*E* = 2000, 0.1, 0.05, 0.025, 0.0153 MPa (from rigid to soft), *v* = 0	—	[23–25]

## Data Availability

The data used to support the findings of this study are available from the corresponding author upon reasonable request.
